The article "Modelling the Potential Impact of Social Distancing on the COVID-19 Epidemic in South Africa" was published in 2020. Journal: Comput Math Methods Med.

# Modelling the Potential Impact of Social Distancing on the COVID-19 Epidemic in South Africa

**DOI:** 10.1155/2020/5379278

**Published:** 2020-10-29

**Authors:** F. Nyabadza, F. Chirove, C. W. Chukwu, M. V. Visaya

**Affiliations:** Mathematics and Applied Mathematics Department, University of Johannesburg, Auckland Park Kingsway Campus, PO Box 524, 2006 Johannesburg, South Africa

## Abstract

The novel coronavirus (COVID-19) pandemic continues to be a global health problem whose impact has been significantly felt in South Africa. With the global spread increasing and infecting millions, containment efforts by countries have largely focused on lockdowns and social distancing to minimise contact between persons. Social distancing has been touted as the best form of response in managing a rapid increase in the number of infected cases. In this paper, we present a deterministic model to describe the impact of social distancing on the transmission dynamics of COVID-19 in South Africa. The model is fitted to data from March 5 to April 13, 2020, on the cumulative number of infected cases, and a scenario analysis on different levels of social distancing is presented. The model shows that with the levels of social distancing under the initial lockdown level between March 26 and April 13, 2020, there would be a projected continued rise in the number of infected cases. The model also looks at the impact of relaxing the social distancing measures after the initial announcement of the lockdown. It is shown that relaxation of social distancing by 2% can result in a 23% rise in the number of cumulative cases whilst an increase in the level of social distancing by 2% would reduce the number of cumulative cases by about 18%. The model results accurately predicted the number of cases after the initial lockdown level was relaxed towards the end of April 2020. These results have implications on the management and policy direction in the early phase of the epidemic.

## 1. Introduction

COVID-19 is an emerging respiratory infection, that is, it is a disease caused by a virus SARS CoV-2 that has not been observed previously in any population or geographic location [1]. It spreads mainly via respiratory droplets produced when an infected person coughs and/or sneezes. The droplets are transferred to another individual through close personal contact such as touching or shaking hands, touching an object or surface with the virus on it, and subsequently touching one's face with contaminated hands [2]. People can also get the infection through breathing in droplets coughed by someone infected [3]. The global spread is increasing and has infected millions, with the highest recorded cases in the USA, Brazil, and India [4–7]. In South Africa, the emergence of COVID-19 was initially influenced by human factors which included international travel to infected countries and consequently local travels, human behaviour, and crowding in cities, among others [8]. Various ways can be used to address, prevent, and combat the spread of COVID-19. These include regular and thorough cleaning of hands with alcohol-based sanitizers, social distancing, avoiding touching one's face, practising good respiratory hygiene, self-isolation, quarantining, restricting travel, and lockdown [3]. There is currently no antiviral treatment or vaccine for COVID-19, and thus, most procedures are just supportive treatment such as the provision of oxygen [8].

The article "Modelling the Potential Impact of Social Distancing on the COVID-19 Epidemic in South Africa" was published in 2020. Journal: Comput Math Methods Med.

In December 2019, a cluster of pneumonia cases was reported in Wuhan, Hubei Province of China, and a novel coronavirus was eventually identified [9]. The first COVID-19 case in South Africa was identified on March 5, 2020, as an imported case from one of the hotspot countries, Italy. The number of imported cases continued to rise in the country until March 17, 2020, when the first locally transmitted cases were identified. At the time of writing, the total number of cases recorded was 85 inclusive of 8 new locally transmitted cases [8]. The new cases came two days after the pronouncement of the national state of disaster by the president of the nation. On March 26, 2020, the nation enforced a 21-day national lockdown to restrict the movement of persons during this period. The restriction largely enforced social distancing a measure to delay and prevent new local and international infections [10]. Social distancing entails limiting close contact with individuals outside the household, in indoor and outdoor spaces [11]. If used effectively, it can delay the time to epidemic peak and reduce the overall number of cases, the number of cases at the epidemic peak, and the total number of severe cases and deaths. The reduction of the number of cases during the epidemic peak and the subsequent spread of cases over a longer time period reduces the burden of health care systems thereby promoting effective case management and treatment [12].

South Africa had about 3,000 (out of about 7,000) critical care beds available between the public and private healthcare sectors reserved for critical COVID-19 patients [13]. A study done in 2017 showed that nationally, there was 1 hospital, 187 hospital beds, and 42 surgical beds per 100,000 population [14]. South Africa had the most number of COVID-19 infections in the whole of Africa, with a total of 2,272 cases as of April 13, 2020. On the same day, there was a total of 1,788,942 cumulative cases and over 117,291 deaths reported worldwide. Of the cumulative cases, 34%, 1%, 52%, 6%, 1%, and 6% were apportioned to the Americas, South-Eastern Asia, Europe, Eastern Mediterranean, Africa, and Western Pacific regions, respectively. The same regions had 25,551, 896, 86,288, 5,364, 501, and 4,181 cumulative deaths, respectively [15]. Receiving over 21 million people annually with the capacity to process up to 28 million, O.R. Tambo International Airport in Johannesburg is Africa's busiest airport. It is not surprising that South Africa's first 77 cases were due to imported cases, with the first 8 local transmissions reported on March 17, 2020. The South African government, however, acted more decisively than most governments around the world by restricting travel from high-risk countries just 9 days after detection of the first local transmission case.

The article "Modelling the Potential Impact of Social Distancing on the COVID-19 Epidemic in South Africa" was published in 2020. Journal: Comput Math Methods Med.

Given that containment of COVID-19 by many countries included lockdown and social distancing, mathematical models that study the transmission dynamics of the pandemic that include the effects of various interventions are of interest [16–23]. These models used the standard or modified SEIR compartmental structure to model the various aspects of COVID-19 dynamics. It is important to note that these models were designed specifically to model the dynamics of the infection for specific countries or regions depending on the level of the epidemic in the affected countries. For instance, [19] presented a modified SEIR model quarantining, death, and protected population compartments to reflect the situation in Italy and [16] presented multiple hosts and reservoirs model for the China situation where the infection is believed to have emanated and introduced into the human population before it spread worldwide. In [21], an individual-based simulation model was used. To quantify social distancing effectiveness, simulation of virus transmission, with and without social distancing measures, was done. In [22], a simple Markov chain model was used to represent the dynamics of COVID-19. The effect of social distancing was implemented by redefining the basic reproduction number on the day measures were implemented to reflect a sufficient decline in how many people each shedding or symptomatic person will infect (i.e., *R*_0_ = 0 is perfect social distancing).

The model considered in this study considers the effect of social distancing on the spread of COVID-19 in South Africa. It resonates with the ideas portrayed in the aforementioned studies. It captures the dynamics of South Africa in the early phase of infection, uses the SEIR structure, uses the public data for COVID-19 data for cumulative cases for South Africa, and incorporates the control measures implemented by the government of South Africa during that phase.

The article "Modelling the Potential Impact of Social Distancing on the COVID-19 Epidemic in South Africa" was published in 2020. Journal: Comput Math Methods Med.

## 2. Methodology

### 2.1. Mobility and the Epidemic Data

The lockdown imposed by the South African government impacted the mobility of citizens significantly. The reduction in mobility meant increased social distancing. So we are concerned with the mobility in South Africa soon after the lockdown. To get a sense of the general pattern of movement of the South African community before and after the lockdown, we use information from Google mobility reports [24].  Figure 1 depicts how visits and length of stay at different places change compared to a baseline (i.e., the median value, for the corresponding day of the week, during the 5-week period March 1 to April 12, 2020). Insights in these reports are created with aggregated, anonymised sets of data from users who have turned on the “location history” settings on their electronic gadgets. The most recent report at the time of writing was until April 12, 2020, and represents data about two to three days in retrospect, the time it takes to produce the reports. Categories that are useful to social distancing efforts, as well as access to essential services, are included in the report. It is evident from Figure 1 that the overall trend in South Africa decreased after the lockdown (March 26, 2020). In particular, the behaviour in retail and recreation (-75%) and grocery and pharmacy (-46%) are similar, particularly a spike just before the lockdown as most people stocked up and did panic-buying, as illustrated in Figure 1(a). In both categories, there were still movements due to essential workers that needed to go to work, with a decrease in activity during weekends. The opposite trends between workplace (-56%) and residential places (+22%) can also be observed, as seen in Figure 1(b). In Figure 1(c), we have the mobility for parks (-58%) and transit stations (-78%).

With regard to the effect of social distancing to the COVID-19 cases, we can also observe from Figure 2 that the number of newly infected cases dramatically decreased after the lockdown, as depicted by the graph of the 7-day moving average. The mobility and epidemic data presents an opportunity to assess the possible impact of social distancing on the progression of COVID-19 in South Africa. In the next section, a mathematical model to perform this assessment is presented.

### 2.2. The Model

We consider an SEIR model where the total population *N* (*t*) at any time *t* is divided into the following compartments: the susceptible population *S*(*t*) composed of individuals with no virus in their system but at risk of contracting the infection when they come into contact with infectious individuals; the exposed population *E*(*t*) comprising of individuals who have the virus but not yet able to transmit the virus through sneezing or coughing; the infectious population *I*(*t*), with either mild or clinical symptoms who can transmit the virus to the healthy individuals resulting in successful infection; and the recovered population *R*(*t*), consisting of individuals who would have recovered either naturally due to robust immune responses or due to supportive treatment available in isolation centres or hospitals. Thus,

(1) $$\begin{array}{c} N\left(t\right)=S\left(t\right)+E\left(t\right)+I\left(t\right)+R\left(t\right). \end{array}$$

COVID-19, as a lower respiratory infection, can be cleared within a few days, and so we shall use the day as the unit of time for our model. The model presented considers COVID-19 infection dynamics over a short period. We, therefore, consider a model for COVID-19 with no vital dynamics as a befitting assumption. As the first cases of COVID-19 in South Africa were due to imported cases, we assume the flow of individuals into South Africa as both susceptible and exposed, since no infectious cases were picked at the entry point but a few days after entry. We assume a constant immigration rate of *Λ*. A proportion *p* (0 < *p* < 1) of the immigrants are assumed to be exposed, and 1 − *p* is assumed to be susceptible. The recruitment rates of *S*(*t*) and *E*(*t*) are therefore (1 − *p*)*Λ* and *pΛ*, respectively. All the imported exposed cases converted into active cases within a minimum of 2 days, and these active cases were the sources of secondary infections in the country. We assume that the new cases were a result of contacts between the susceptible individuals *S*(*t*) with the proportion of infectious individuals, *I*(*t*)/*N*(*t*). The effective contact rate is *β*, giving a force of infection *λ* = *β* (*I*(*t*)/*N*(*t*)), and the number of new infections out of *S*(*t*) and into *E*(*t*) as *βI*(*t*)*S*(*t*)/*N*(*t*). The exposed cases progress to active cases between 2 and 14 days at a constant progression rate *κ* giving the number of individuals moving out of *E*(*t*) and into *I*(*t*) as *κE*(*t*). The infectious individuals are assumed to recover at a constant rate *σ*. The total number of recovered individuals moving out of *I*(*t*) into *R*(*t*) is given by *σI*(*t*). Currently, there is no evidence of reinfection after recovery in South Africa, and hence, we assume that no recovered individual can become susceptible to the infection.

The article "Modelling the Potential Impact of Social Distancing on the COVID-19 Epidemic in South Africa" was published in 2020. Journal: Comput Math Methods Med.

South Africa implemented a national lockdown on day 21 since the announcement of the first case, where day 1 is March 5, 2020. The lockdown saw the complete blockage of imported cases, and hence, the infection after day 21 was driven by the imported cases which were already in the country until day 21 and the local cases which resulted from these imported cases. After day 21, there were no more recruitments into the susceptible and exposed populations due to immigration as a result of the lockdown. This is tantamount to setting both *Λ* and *p* to zero after day 21. We represent the recruitment rate *S*_rec_ of imported susceptibles by

(2) $$\begin{array}{c} S\text{rec}=\left\{\begin{array}{c} \left(1-p\right)\Lambda ,t_{0}\leq t<t_{\text{lock}},\\ 0,t\geq t_{l\text{ock}}, \end{array}\right. \end{array}$$

where *t* = *t*_0_ is the time in which the first infectious case was identified and *t* = *t*_lock_ is the time in which the lockdown was effected. In our model, *t*_0_ = 0 and *t*_lock_ = 21. Similarly, the recruitment rate *E*_rec_ of the exposed population is given by

(3) $$\begin{array}{c} E\text{rec}=\left\{\begin{array}{c} p\Lambda ,t_{0}\leq t<t_{\text{lock}},\\ 0,t\geq t_{\text{lock}}. \end{array}\right. \end{array}$$

At the inception of the lockdown, the main mitigation strategy against the pandemic was social distancing between individuals. Social distancing reduces the contact rate between infectious and susceptible individuals. We incorporate social distancing through a constant rate *ρ* (0 < *ρ* < 1), where *ρ* 0 means that the social distancing is near perfect, and *ρ* 1 means there is no social distancing. We assume that *ρ* does not assume its extreme values since the locking down in its inherent nature enforces some social distancing, and due to the nature of the settlement patterns in some parts of South African suburbs and the socialisation of family units, perfect social distancing is not attainable. The force of infection is modified as follows:

(4) $$\begin{array}{c} \lambda =\left\{\begin{array}{cc} \;\frac{\beta I}{N}, & \;t_{0}\leq t<t_{\text{lock}},\\ \frac{\rho \beta I}{N}, & t\geq t_{\text{lock}}. \end{array}\right. \end{array}$$

The model diagram is presented in Figure 3.

The system of differential equations capturing the assumptions on COVID-19 for South Africa before and after the lockdown is presented in (5) and given by

(5) $$\begin{array}{c} \frac{dS}{dt}=S_{\text{rec}}-\lambda S, \end{array}$$

(6) $$\begin{array}{c} \frac{dE}{dt}=E_{\text{rec}}+\lambda S-\kappa E, \end{array}$$

(7) $$\begin{array}{c} \frac{dI}{dt}=\kappa E-\sigma I, \end{array}$$

(8) $$\begin{array}{c} \frac{dR}{dt}=\sigma I, \end{array}$$

subject to the following initial conditions

(9) $$\begin{array}{c} S\left(0\right)=S_{0}>0,\;E\left(0\right)=E_{0}\geq 0,\;I\left(0\right)=I_{0}\geq 0,\;R\left(0\right)=R_{0}\geq 0. \end{array}$$

Using the next-generation matrix method as in [25, 26], the basic reproduction number *ℜ*_0_ of the model system (5) is determined where

(10) $$\begin{array}{c} F=\left(\begin{array}{cc} 0 & \beta \\ 0 & 0 \end{array}\right)\text{and }V=\left(\begin{array}{cc} \kappa & 0\\ -\kappa & \sigma \end{array}\right). \end{array}$$

The product of *FV*^−1^ is given by

(11) $$\begin{array}{c} FV^{-1}=\left(\begin{array}{cc} \frac{\beta }{\sigma } & \frac{\beta }{\sigma }\\ 0 & 0 \end{array}\right) \end{array}$$

with the spectral radius denoted by

(12) $$\begin{array}{c} \nu \left(FV^{-1}\right)=R_{0}=\left\{\begin{array}{c} \;\frac{\beta }{\sigma },t_{0}\leq t<t_{\text{lock}},\\ \frac{\rho \beta }{\sigma },t\geq t_{\text{lock}}. \end{array}\right. \end{array}$$

The article "Modelling the Potential Impact of Social Distancing on the COVID-19 Epidemic in South Africa" was published in 2020. Journal: Comput Math Methods Med.

## 3. Results

### 3.1. Data and Parameter Estimation

The epidemic data was obtained from [27] and the information released through the South African government newsroom [28]. According to Statistics South Africa [29], the midyear population estimates for 2019 showed that the country's population stood at 58,775,022. This statistic is important in estimating the number of susceptible individuals at the start of the epidemic. It is important to note that at the beginning of the epidemic, the entire country is considered to be naive as the index cases were all as a result of individuals who travelled to places that had already ongoing epidemics such as Asia, Europe, and North America. The first case of COVID-19 in South Africa is reported to have travelled to Italy with his wife (as a part of a group of 10) and had returned on March 1, 2020 [8]. The data on COVID-19 in this study was mainly obtained from the media releases by the South African government [28] and the National Institute of Communicable Diseases [8] from March 5 to April 13, 2020. The data included the daily updates on the cumulative numbers of COVID-19 cases and their distribution per province. The number of cumulative cases used for our simulations is available at the data repository and newsroom [27, 28]. The formulated model is then fitted to the data in two epochs, viz., the period before the lockdown and the duration after the lockdown. The uniqueness of this model is that it considers a constant daily influx of people into South Africa with a proportion of those coming into the country having been exposed to COVID-19. After the lockdown, the constants that model the movement of people into the country are then set to zero, and then, the epidemic is assumed to be mainly driven by local transmission dynamics.

We fit the model to the data recorded before the lockdown using the least-squares curve fitting method in Matlab. Parameter bounds are set based on recent work on the epidemic in countries such as China [30–33], Korea [34, 35], and Italy [36]. The reproduction numbers of COVID-19 were determined from various mathematical models for the epidemic in China [33, 37–40]. Given the known values of the incubation period, 1/*k*, and the duration of infectivity, 1/*σ*, we estimate the effective contact rate *β*, for the current epidemic in South Africa. The parameter values are given in Table 1.

The article "Modelling the Potential Impact of Social Distancing on the COVID-19 Epidemic in South Africa" was published in 2020. Journal: Comput Math Methods Med.

### 3.2. Sensitivity Analysis

The SEIR model (5) has some limitations especially on determining the parameter values. The various processes driving the model dynamics have several complexities, and hence, the model parameters are best measured approximately. The parameters have substantial variations depending on the geographical region, demographic factors, settlement patterns, and several other factors. Besides, some of the parameters may just be stochastic. The model thus has inherent epistemic uncertainty which results from a lack of knowledge about the value of parameters which are then assumed to be constant throughout the model analysis [42]. To adapt the model simulations to the South African scenario, we first used parameter values from other regions, fitted the model to the daily cumulative cases, and obtained the best fit values of the parameters. To cater to the inherent complexities around these best-fit values, we use the Latin Hypercube Sampling (LHS) technique for uncertainty quantification and sensitivity analysis. This is a reliable and efficient technique for the detection of such epistemic uncertainties allowing unbiased estimates of the average model output with fewer samples than other sampling methods to achieve the same accuracy. To measure the strength of the relationship between each input variable and each output variable, the LHS technique is combined with the partial rank correlation coefficients (PRCCs) [43]. We use Figures 4(a) and 4(b) to show the contribution of different parameters before and after the lockdown. Their contribution is measured against the number of cumulative cases in South Africa. The range of values used is given in Table 1.  Figure 4(a) shows that the immigration parameters *p* and *Λ* are strongly positively correlated to the number of cumulative cases before the lockdown. This means that the increase in the proportion of exposed immigrants and the rate of immigration is associated with the increase in cumulative cases.  Figure 4(b) shows that the infection parameter *β* and the social distancing parameter *ρ* are strongly positively correlated to the cumulative cases whilst the infection progression and recovery parameters *κ* and *σ* are strongly negatively correlated to the cumulative cases after lockdown. The increase in the infection rate and the increase in the social distancing parameter (i.e., decreasing social distancing level) is associated with the increase in cumulative parameters whilst the increase in the progression and recovery rates is associated with the decrease in cumulative cases.

The article "Modelling the Potential Impact of Social Distancing on the COVID-19 Epidemic in South Africa" was published in 2020. Journal: Comput Math Methods Med.

### 3.3. Model Fitting and Simulations

In this section, we fit the designed model to the cumulative cases of South Africa before the lockdown (see Figure 5) in the absence of any intervention to obtain the best fit model parameter values for the South African dynamics. We present the model simulations with these best fit parameter values to predict the likelihood of occurrence of the peak number of cases had the lockdown not been effected at day 21 (Figures 6 and 7). We also fit the model to the cumulative cases when lockdown and social distancing (Figure 8) were effected to obtain the best-fit parameter values. We use the resulting fit to make possible predictions of the potential impact of different levels of compliance to social distancing with the lockdown in place (Figure 9).

Figure 5 shows that the model (5) fits well to the cumulative cases of South Africa, and the best fit parameter values are the current model values that could be used for prediction in the absence of intervention. Using the best-fit parameter values, Figure 6 shows that the peak of cumulative cases would have been reached in mid-May before the number of cases begins to decline.  Figure 7 is an extract of Figure 6 showing the number of exposed and infectious populations in the absence of any intervention. The figure shows that there would be more infectious cases at the peak than the exposed cases by the time the peak is reached.

Figure 8 shows that the model (5) fits well with the cumulative cases of South Africa up to April 13, 2020, in the presence of the intervention, and the best-fit parameter values are the current model values that could be used for prediction in the presence of intervention. We note that the best fit for social distancing after lockdown is about 55% (*ρ* = 0.45).  Figure 9 shows the COVID-19 model fitting and predictions for the cumulative infected cases for various levels of social distancing. The simulations show that if the level of social distancing is maintained at 55%, then the number of cumulative cases will continue to grow exponentially. Reducing the level of social distancing from 55% to 53% (*ρ* = 0.47) would increase the number of cumulative cases by about 23% at the end of lockdown on April 30, 2020. Increasing the level of social distancing from 55% to 57% (*ρ* = 0.43), 59% (*ρ* = 0.41), and 61% (*ρ* = 0.39) would avert the cumulative cases by about 18%, 32%, and 53%, respectively, at the end of the lockdown on April 30, 2020. Our model fitting and predictions suggest that the current level of social distancing as of 13 April 2020 under lockdown for South Africa is not good enough to flatten the curve, and any relaxation from this will lead to a spike in the cumulative cases. The predictions also suggest that efforts to realise the flattening of the curve should be sustained at least at 60% (*ρ* = 0.4) level of social distancing by the time the lockdown ends on April 30, 2020.

The article "Modelling the Potential Impact of Social Distancing on the COVID-19 Epidemic in South Africa" was published in 2020. Journal: Comput Math Methods Med.

## 4. Conclusion

There has been a huge demand for research to quantify the control measures instituted by many countries to contain COVID-19 globally. Understanding the impact of these control measures requires knowledge and expertise drawn from various scientific disciplines including mathematical modelling. The role of mathematical models' insights formed the national response to the pandemic in South Africa. The idea of social distancing was to flatten the epidemic growth curve, thus allowing time to prepare for the worst-case scenarios, and was drawn from mathematical models for the COVID-19 epidemic. This was critical in preventing the overwhelming of health care facilities and minimising the number of deaths.

We presented a deterministic model to assess the impact of social distancing on the transmission dynamics of COVID-19 in South Africa taking into account the initial imported cases before the lockdown in the early phase of the pandemic. The model fitted well to data with a reproductive number of 2.5 at the initial phase of the pandemic. The fitting generated the estimated COVID-19 transmission rates for South Africa. The insights gained from the current study contributed to the current levels of interventions using social distancing in South Africa.

The quantification of the levels of social distancing was significant in deciding the easing of lockdown regulations. The lockdown period had an estimated social distancing parameter of around 0.54.

This means that in spaces that accommodated an average of a hundred people, only fifty should be allowed to control the pandemic. The role played by immigration was also crucial in the growth of the pandemic especially in March 2020 before the closure of South African borders. The results suggest that individuals migrating into South Africa played an important role in driving the infection in South Africa, and the prevention of infections happening elsewhere on the globe needs special attention due to improved mobility of humans. Particular attention needs to be focused on travellers beyond the lockdown to ensure that screening is effectively done when travellers enter the country.

The article "Modelling the Potential Impact of Social Distancing on the COVID-19 Epidemic in South Africa" was published in 2020. Journal: Comput Math Methods Med.

The sensitivity results show the shift in the drivers of infection before and after the implementation of interventions. This may imply that any intervention leads to emerging challenges due to shifting in the drivers, and hence, proper planning is needed to scale up efforts to avert any emerging issues. Since all the parameters after lockdown have a strong correlation to the number of cumulative cases, holistic strategies are required to reduce the processes that increase the number of cases simultaneously with those decreasing the number of cumulative cases.

The current levels of social distancing were predicted to be inadequate especially during the initial stages of the pandemic with exponential growth in the number of cases. There is a need for more aggressive and robust multicontrol approaches that target the reduction of the infection rate, an increase of social distancing levels, rapid detection of exposed cases, and increase in the recovery of active cases. The shifting in drivers of infection after implementation of lockdown imposed threats to the preparedness of the South African health care system in the aftermath of the lockdown. The use of multidisciplinary collaboration and predictive tools is needed to forewarn the South African health care system of such shifts and enhance emergency preparedness responses.

Given that the research was done between March 5 and April 13, 2020, the current scenario of the epidemic of September 30, 2020, depicts an epidemic that has passed its peak with the recorded numbers of new cases on the decline. A decline in the number of reported deaths also declined significantly. Fears however remain on the possibility of the second wave of the epidemic as has been observed in Spain, the United Kingdom, Australia, and Serbia.

The model presented here is not without shortcomings. The dynamics of COVID-19 combined with the economic and social dynamics of South Africa present a complex scenario from a modelling perspective. On the social dynamics, social distancing in many of the informal settlements has been difficult to enforce due to the high density of people. In addition, the economic dynamics in many of the informal settlements is influenced by informal trading, thus creating difficulties and hardships to people during a lockdown. There were relaxations of the social distancing measures after the lockdown to mitigate the economic and social challenges of the general population. These relaxations had the potential to dilute the intended effects of social distancing. The model presented in this paper was simple and did not capture these complexities. Despite the shortcomings, the results present some interesting results in which even after the simulations, the data that was released on the epidemic still fell within the predictions of the model.

The article "Modelling the Potential Impact of Social Distancing on the COVID-19 Epidemic in South Africa" was published in 2020. Journal: Comput Math Methods Med.

## Figures and Tables

**Figure 1:** Google mobility report for South Africa from March 1 to April 12, 2020, for (a) retail and recreation, and grocery and pharmacy, (b) workplace and residential, and (c) parks and transit stations.

**Figure 2:** A decrease in newly infected cases (%) since the lockdown, together with a 7-day moving average, for the 40 data points.

**Figure 3:** Model diagram for COVID-19 for South Africa with immigration, lockdown, and social distancing.

**Figure 4:** (a) Influence of parameter values on the cumulative cases before the lockdown. (b) Influence of parameter values on the cumulative cases after the lockdown.

**Figure 5:** Model fit to data for COVID-19 before the lockdown. The best-fit parameter values are as follows: *Λ* = 11244, *p* = 1.7598 × 10^−5^, *β* = 1.1411, *κ* = 0.655, *σ* = 0.4482, and *ρ* = 1.

**Figure 6:** A simulation model for the SEIR model for all the populations in the absence of any intervention, i.e., *ρ* = 1. The best fit parameter values are as follows: *Λ* = 11244, *p* = 1.7598 × 10^−5^, *β* = 1.1411, *κ* = 0.655, and *σ* = 0.4482.

**Figure 7:** A simulation model for the SEIR model for exposed and infected in the absence of any intervention, i.e., *ρ* = 1. The best-fit parameter values are as follows: *Λ* = 11244, *p* = 1.7598 × 10^−5^, *β* = 1.1411, *κ* = 0.655, and *σ* = 0.4482.

**Figure 8:** The graph shows COVID-19 model fitting for the cumulative infected cases for South Africa before and after lockdown. The red dots are the cumulative reported number of COVID-19 cases before and after lockdown. The red vertical line represents the start of the national lockdown. The continuous curve represents the model fit. The best-fit parameter values are as follows: *Λ* = 11244, *p* = 1.7598 × 10^−5^, *β* = 1.1411, *κ* = 0.655, *σ* = 0.4482, and *ρ* = 0.453. Note that *ρ* = 0.453 represents about 55% compliance in social distancing.

**Figure 9:** The graph shows COVID-19 model fitting for the cumulative infected cases for various scenarios. The trajectories for different levels of social distancing are shown by the different line types. The red dots are the cumulative reported number of COVID-19 cases in South Africa before the lockdown and two weeks after the lockdown. The red vertical line denotes the time when a lockdown was implemented by the government with a delay of one data point as the reported cases represent posterior data. The best-fit parameter values are as follows: *Λ* = 11244, *p* = 1.7598 × 10^−5^, *β* = 1.1411, *κ* = 0.655, *σ* = 0.4482, and *ρ* = 0.453.

The article "Modelling the Potential Impact of Social Distancing on the COVID-19 Epidemic in South Africa" was published in 2020. Journal: Comput Math Methods Med.

**Table 1:** Parameters of the SEIR model for South Africa and their values.

Symbol	Parameter description	Value (range)(day^*−*1^)	Source
*β*	Effective contact rate	1.0598 (0.9011-1.400)	Data fit
*k*	Progression rate	0.5 (0.2-0.6)	[35]
*σ*	Recovery rate	0.4345 (0.2-0.5)	[33, 35]
*ρ*	Social distancing parameter	(0, 1)	By definition
*p*	Proportion of exposed immigrants	(0, 1)	By definition
*Λ*	Daily rate of immigration	11 244 (10 000-25 000)	[41]

## Data Availability

The data used in this study is available in https://github.com/dsfsi/covid19za/tree/master/data.
